The article "TrustBlock: An adaptive trust evaluation of SDN network nodes based on double-layer blockchain" was retracted in 2025. Reasons: compromised peer review; unreliable results or conclusions; concerns about the peer review.

# TrustBlock: An adaptive trust evaluation of SDN network nodes based on double-layer blockchain

**DOI:** 10.1371/journal.pone.0228844

**Published:** 2020-03-10

**Authors:** Bo Zhao, Yifan Liu, Xiang Li, Jiayue Li, Jianwen Zou

**Affiliations:** Key Laboratory of Aerospace Information Security and Trusted Computing, Ministry of Education, School of Cyber Science and Engineering, Wuhan University, Wuhan, China; University College London, UNITED KINGDOM

## Abstract

The data layer devices in the Software Defined Network (SDN) play an important role in packet forwarding. However, whether the forwarding task can be efficiently completed by the node has not attracted enough attention. A method called TrustBlock is proposed in this paper, which introduces trust as a security attribute in SDN routing planning. Besides, in order to enhance the integrity and controllability of trust evaluation, the double-layer blockchain architecture is established. In the first layer, the behavior data of the node is recorded, and then the trust calculation is performed in the second layer. In the evaluation model, nodes’ trust is calculated from three aspects: direct trust, indirect trust and historical trust. Firstly, from the perspective of security, blockchain is used to achieve identity authentication of nodes, after that, from the perspective of reliability, the forwarding status is used to calculate the trust value. Secondly, consensus algorithm is used to filter malicious recommendation trust value and prevent colluding attacks. Finally, the adaptive historical trust weight is designed to prevent the periodic attack. In this paper, the entropy method is used to determine the weight of each evaluation attribute, which can avoid the problem that the subjective judgment method is not adaptable to the weight setting. Simulation results show that the detection rate of the TrustBlock is up to 98.89%, which means this model can effectively identify the abnormal nodes in SDN. Moreover, it is attractive in terms of integrity and controllability.

## 1. Introduction

Through centralized control of network devices, Software Defined Network (SDN) provides a flexible, dynamic and automatic network configuration, and has been widely used in the various scenarios, such as Internet of things (IoT), cloud computing, edge computing, etc. For instance, in the IoT environment, the network knowledge map can be improved through the centralized control, and in addition, a policy-based, automatic, large-scale and complex network control can be achieved through SDN. Therefore, make the IoT network easier to manage. Security threats can be found and addressed more easily by modifying the transparency of traffic provided to the edge of the network.

With the development and application of SDN, the deficiency of itself to deal with security threats has gradually emerged [1]. The data layer devices receive instructions from the controller through the southbound interface and complete specific network data processing according to these instructions. Meanwhile, the network configuration and runtime state information are collected by the SDN data layer devices and transformed to the controller. Once the data layer device is attacked, the network data processing speed will slow down or the network even fails to complete the normal packet forwarding task. In addition, attackers may take advantage of the network state information to launch attacks. In a conclusion, SDN data layer equipment security is very important. However, at present, most researchers focus on DoS/DDoS attacks and forwarding path planning in SDN [2–9]. How to ensure the nodes’ trust situation and the security of SDN data layer device is the focus in this paper.

At present, the attacks on SDN data layer can be divided into external attacks and internal attacks. External attacks include information interception, information monitoring, node masquerading, DoS/DDoS attacks and so on. The attacker cannot dominate the network node. Therefore, the traditional security mechanisms such as access control, intrusion detection, and authentication mechanism can resist and respond the attack effectively. Internal attacks are initiated by attackers who have captured and cracked the normal node, including packet discarding, information retransmission and stealing, publishing false data packets and so on. Compared with external attacks, internal attacks are more covert and difficult to detect. It is difficult to defend internal attacks using only traditional security technology. Trust mechanism can identify malicious nodes and selfish nodes and resist network intrusion, which is an effective supplement to traditional security measures.

Based on the above problems, trust is introduced as a security attribute to evaluate the SDN data layer devices in this paper. In the process of node interaction, there are problems such as uncertainty, uncontrollability, ambiguity and incompleteness. Trust can help the controller better understand the node status, reduce the risk of node interaction, and enhance the robustness of SDN system. In practical applications, SDN controller and all its subordinate data layer devices (such as switches) constitute a management domain, and devices can cooperate within or across domains to achieve specific requirements. Domain managers need to establish, evaluate and update trust relationships between each other, and devices in the network also need to dynamically adjust and update trust relationships with others. Nowadays SDN often rely on the inherent trust, which may be used by attackers for security intrusion. Assessing the trust values between nodes is an effective strategy. The trust value can be regarded as the security attribute of route planning.

According to "trust ≈ security + reliability", the trust evaluation model consists of reliability and security, and the comprehensive trust is made up of three parts: direct trust, indirect trust and historical trust. Considering the fixed energy supply and storage capacity of devices in data layer, the blockchain is introduced to realize safe and effective trust value storage and sharing. Blockchain is a new and attractive data storage technology with distributed consensus, tamper-proof and undeniably features. The traceability of blockchain is used to realize the authentication of nodes and tracking of malicious nodes, the consensus mechanism of blockchain is used to filter malicious recommendation nodes and prevent collusive attack, and the immutability of blockchain is used to realize the storage of trust value.

The contributions of this paper mainly include the following aspects:

1. Trust evaluation is combined with blockchain to reduce the influence of malicious nodes. Avoid the extra overhead of adding hardware
2. Using entropy method to determine the weight of each evaluation attribute, avoiding the problem that the subjective judgment method is not adaptable to the weight setting, and ensuring the validity and objectivity of the decision.
3. Users don't need to care about the trust management process. Using nodes with high trust values can obtain more reliable services and enhance network availability.

The rest of the paper is organized as follows. Section 2 reviews related work. Section 3 and 4 present a brief design of the TrustBlock and the double-layer blockchain architecture. The calculation details of the trust value are shown in Section 5. Section 6 shows the experimental results and then concludes them in Section 7.

## 2. Related work and blockchain

### 2.1. Related work

For the malicious node problem in data layer, the main method is using the authorization authentication mechanism to prevent malicious nodes from accessing the network. In [10], the author proposed a method called AuthFlow, an authentication and access control mechanism based on host credentials. Othman et al. [11] proposed a hybrid control security model and designed a new signature algorithm based on TLS to protect the whole communication process of SDN. However, these methods require a centralized trust management module and add signature and authentication load, which have an impact on system performance.

For the failure node problem in data layer, the main method is using the fast recovery mechanism to recover the failed node through the entire network information. Specifically, it mainly includes the following steps: (1) When one device fails, other devices detect problems and report to the controller. (2) SDN controller calculates the rules according to the historical information. (3) SDN controller sends the calculated results to the affected network nodes in the data layer. (4) Affected devices update their flow tables. This method is a recovery strategy after the accident has occurred, which will affect the data transmission efficiency. If the node trust can be evaluated in the SDN and a more reliable node can be selected for data transmission, the unnecessary losses can be reduced.

### 2.2. Blockchain

The blockchain originated from the digital currency bitcoin, which is a shared distributed database technology, and its advantages are mainly reflected in three aspects: decentralization, traceability and immutability. Researchers have proven that blockchain can be applied to a variety of scenarios. In the field of IoT, IBM developed Adept with blockchain to address the problem of centralized management. Adept can not only ensure the normal communication of intelligent devices, but also record the operation status of devices in real time, facilitating the tracking and maintenance of failed devices. In the field of network communication, KSI [12] used blockchain to provide underlying security for SDN, and the communication service provider used blockchain to provide data communication and management services, including some core operations [13]. In the field of cloud storage, Storj [14] was developed based on blockchain, which achieve low cost while ensuring security. Not only is the Storj’s reliability comparable to high-end cloud storage products, but also the cost is only 1–2% of traditional cloud storage. These applications are enough to demonstrate the great development potential of blockchain, which is used in this paper to realize the node trust evaluation of SDN.

## 3. Overview of TrustBlock

This paper proposes a trust evaluation mechanism of SDN named TrustBlock to solve the above problems. As shown in Fig 1, the participating entities including users, SDN and verifiers. When the SDN works, the user inputs the data packets to start the forwarding task. The data layer device in SDN contains hardware-based and software-based network nodes. The double-layer blockchain represents the storage location of trust value, which occupies some node space in the data layer, and is divided into two layers: node behavior data block and node trust data block. Any user (including new authorized user, historical user or SDN administrator, etc.) who wants to access the trust value of SDN data layer device is classified as verifier, and any verifier has the right to view the trust value of any node at any stage.

**Fig 1:** Overview of TrustBlock.

In SDN, trust is obtained through observation of evaluation nodes and recommendation of third-party nodes. The trust value of a node is not fixed, and will change over time depending on the behavior of the node. As shown in Fig 2, node *i* is the node to be evaluated, and node *j* is the direct communication node of *i*, node *k*1, *k*2 and *k*3 are neighbor nodes within the common communication range of node *i* and *j*. Node j can directly evaluate node *i*, and indirectly evaluate through neighbor nodes. By combining the historical trust value, the comprehensive trust value of node *i* can be finally obtained. Based on this, the comprehensive trust (*CTrust*) of nodes is calculated from three aspects of direct trust (*DTrust*), indirect trust (*ITrust*) and historical trust (*HTrust*).

**Fig 2:** Relationships between SDN nodes.

Node trust evaluation of SDN is affected by multiple factors. Establishing node trust system is the premise and basis of computing node trust. According to the “trust ≈ security + reliability” [15], a comprehensive SDN node trust evaluation system should be established by combining reliability and security. The final node trust evaluation system is shown in Fig 3. Considering that normal nodes also have poor transmission quality due to cache overflow or poor link quality, trust evaluation is conducted after a period (for example, 10 minutes). The trust of node *r*_*i*_ at time *t* can be expressed as:

$${CTrust}_{i}(t)=\omega_{1}\times {DTrust}_{i}(t)+\omega_{2}\times {ITrust}_{i}(t)+\omega_{3}\times {HTrust}_{i}(t),$$ (1)

**Fig 3:** TrustBlock trust evaluation system.

To better describe the trust model in this paper, the definitions are as follows:

1. Trust. Trust can be described as Trust = (A, L, V). In the process of calculating the trust value of SDN nodes, A = {a_1_, a_2_, …, a_n_} is expressed as a set of trust evaluation attributes. a_k_(1 ≤ k ≤ n) is expressed as a description of the k-th attribute, such as task completion, node transfer rate, data conversion rate, etc. L = {l_1_, l_2_, …, l_k_} is expressed as a fuzzy set of trust evaluation degree, which can be divided according to the needs of users. For the convenience of representation, the node trust level is divided into {0, 1, 2, 3} in this paper, which means {not trusted, generally trusted, relatively trusted, very trusted}. V = {v_1_, v_2_, …, v_n_} is expressed as a trust evaluation vector, v_k_(1 ≤ k ≤ n) is expressed as the value of the corresponding attribute a_k_.
2. Direct trust. Direct trust is expressed as the node trust directly obtained from the node's behavior in a given context. The direct trust of node *r*_*i*_ at time t can be expressed as *DTrust*_*i*_(*t*).
3. Indirect trust. Indirect trust refers to the value of trust that is not got from direct communication but from third-party recommendations. The indirect trust of node *r*_*i*_ at time t can be expressed as *ITrust*_*i*_(*t*).
4. Historical trust. In order to prevent malicious nodes from using the continuous normal behavior to quickly improve the trust value, the historical trust is introduced into the evaluation model. The historical trust of node *r*_*i*_ at time t can be expressed as *HTrust*_*i*_(*t*).
5. Weights. W = {*w*_1_, *w*_2_, …, *w*_*n*_} is expressed as a set of weights for each evaluation attribute. *w*_*k*_(1 ≤ k ≤ n) indicates the relative importance degree of the corresponding attribute *a*_*k*_. The *ω*_1_, *ω*_2_, *ω*_3_ can be obtained by adding the weights of the corresponding evaluation attributes. In order to ensure the validity and objectivity of trust evaluation, the entropy method is used to calculate the weight of each evaluation attribute.

Assume that the SDN contains *m* evaluation nodes and *n* evaluation attributes, the value matrix is got of each trust evaluation attribute as $X=[\begin{array}{ccc} x_{11} & \cdots & x_{1n}\\ \vdots & \ddots & \vdots \\ x_{m1} & \cdots & x_{mn} \end{array}]$. *x*_*ij*_ represents the value of the *j-th* evaluation attribute for the *i-th* node. In order to reduce the impact of outliers on the evaluation matrix, the nodes with large fluctuations is removed. The calculation process is as follows.

- Normalize the matrix. The positive indicator and the negative indicator represent different meanings, so different algorithms are used to standardize the data. The specific algorithm is as follows:
  For positive indicators:
  $$x_{ij}^{\prime }=\frac{x_{ij}-min\{x_{1j},\ldots ,x_{mj}\}}{\text{max}\left\{x_{1j},\ldots ,x_{mj}\right\}-min\{x_{1j},\ldots ,x_{mj}\}},$$ (2)
  For negative indicators:
  $$x_{ij}^{\prime }=\frac{max\left\{x_{1j},\ldots ,x_{nj}\right\}-x_{ij}}{max\left\{x_{1j},\ldots ,x_{nj}\right\}-min\left\{x_{1j},\ldots ,x_{nj}\right\}},$$ (3)
  For convenience, the normalized data is still recorded as *x*_*ij*_.
- Calculate the entropy value. By calculating the proportion of the *j-th* trust evaluation attribute with the *i-th* node, the entropy value of the *j-th* trust evaluation attribute *e*_*j*_ can be obtained:
  $$e_{j}=-k\sum_{i=1}^{m}\frac{x_{ij}}{\sum_{i=1}^{n}x_{ij}}ln\left(\frac{x_{ij}}{\sum_{i=1}^{n}x_{ij}}\right),\;i=1,\ldots ,m,j=1,\ldots ,n,$$ (4)
  k = 1/ln(n) > 0, which means *e*_*j*_ ≥ 0
- Calculate the weight value. By calculating the entropy redundancy of each attribute, the weight of each indicator *w*_*j*_ is obtained.
  $$w_{j}=\frac{1-e_{j}}{\sum_{j=1}^{n}\left(1-e_{j}\right)},\;j=1,\ldots ,n,$$ (5)
  Get weight W = {w_1_, w_2_, …, w_n_}.

The detailed calculation method of each part is introduced in the following sections.

## 4. Double-layer blockchain architecture

Traditional network system's node trust is scattered and isolated. The trust value of a node in one network system cannot be shared with another system. With the development of the Internet, the relationship between different networks gradually strengthens, especially in the SDN. With the expansion of the network scale, the complexity of the message interaction between the controller and the switch is getting higher and higher. In order to prevent control congestion caused by excessive controller load, the existing SDN mostly realizes domain management of the network through multi-controller scheme. Regarding the cross-domain cooperation of nodes in SDN, if the trust information of nodes can be shared among various domains, it will bring great convenience to node management. Blockchain makes it possible to share trust value in safety.

Blockchain can guarantee the integrity and controllability of node trust evaluation model, but time-intensive main block election task may lead to high confirmation delay of data storage. In order to improve efficiency, a double-layer blockchain is designed, the first layer records data and the second layer performs Proof of Work (PoW) consensus algorithm in the background.

The first layer is the node behavior data block to ensure that the behavior of nodes can be traced back, and the nodes cannot deny the behavior that has taken place. The node behavior data block architecture is shown in Fig 4, each block is anchored to the blockchain with a merkle root, which is generated by the hash algorithm, and the hash function has the characteristics of anti-collision. Any modification behavior can change the value of merkle root, which means that the node behavior can be traced and cannot be tampered with. Node behavior data block contains important information for analysis such as node number, node digital signature, a large amount of node behavior data and timestamp.

**Fig 4:** Node behavior data block structure.

In order to reduce the time overhead, when the first layer is performing data processing, the second layer performs the main block election task synchronously in the background, and completes the calculation of the trust value. The node trust data block architecture is shown in Fig 5, includes direct trust, indirect trust, historical trust and comprehensive trust, which protect the trust value of nodes from tampering and supervise the behavior of nodes in the network. The trust value of the node can be viewed by all verifiers.

**Fig 5:** Node trust data block structure.

The overall structure of the double-layer blockchain is shown in Fig 6. Node behavior data block from the first layer to store specific node behavior data. Node trust data block from the second layer to store node trust value. Once the suspicious node is found, it will be immediately marked to set access rights or prohibit from joining the SDN. Trust evaluation system uses mathematical theory and methods to model node behavior. Due to the randomness, fuzziness and complexity of the behavior of nodes in the SDN, the fuzzy comprehensive evaluation method is used to analyze the trust attribute.

**Fig 6:** Two-layer blockchain structure.

There are three stages in TrustBlock construction: node behavior data block establishment, consensus achievement and trust computing, and node trust data block establishment. The detailed process is described in section 5.

## 5. Calculation of trust value

### 5.1 Direct trust

In a given context, the node trust value obtained by the node's direct communication behavior is called direct trust. In this paper, the fuzzy comprehensive evaluation model is used to analyze the trust attribute. It mainly includes the following steps:

#### 5.1.1 Evaluation attributes set

Trust evaluation attributes are selected from the perspectives of reliability and security, the factors are expressed as follows:

From the aspect of security, blockchain is used to realize node identity authentication. Attacks can be accomplished by modifying packet data or injecting additional packets. In order to ensure that the data received is reliable, it is necessary to identify whether the node is legitimate. The blockchain uses the public-private key pair to identify the nodes’ identity.

Node identification key pair (*PK*_*i*_, *SK*_*i*_): public-private key pair is the identity certificate of node *i*, *SK*_*i*_ is used to sign the packet, *PK*_*i*_ is used for verification. Before the forwarding task, the node's identity information is first verified. If the validation is successful, the received data will be forwarded. If the validation is failure, the trust degree of the node is directly determined to be 0, and the node is considered to be untrusted, which will be refused to join the SDN.

After node authentication is successful, the node's running status is analyzed from the perspective of reliability, including the following attributes:

$$Task\_Completion=1-\frac{{data}_{in}-{data}_{out}}{{data}_{in}},$$ (6)

*Task*_*Completion* represents the percentage of data transmitted successfully. The closer *Task*_*Completion* is to 1, the more stable the node running state is and the lower the packet loss probability is.

$$Transfer\_rate=\frac{{data}_{transfer}}{time},$$ (7)

*Transfer_rate* represents the amount of data transmitted per unit time, which is the main attribute to measure the transmission capacity of a node.

$$Conversion\_rate=\frac{{data}_{forward}}{{data}_{in}},$$ (8)

*Conversion_rate* indicates the ratio of the forwarded data to the received data at the same time. The higher *Conversion_rate* is, the more efficient the node is.

$$Repetion\_rate=\frac{{data}_{repeat}}{{data}_{out}},$$ (9)

*Repetion_rate* indicates the ratio of duplicate packets to transmitted packets. If there are a large number of packets with the same content, the node may be carrying out repeated attacks intended to consume network resources. The lower *Repetion_rate* is, the less content is repeatedly sent.

*Node_Resource* indicates the remaining resource of the node. When the user's demand for network resources (such as link bandwidth, storage space, processor capacity, etc.) exceeds the remaining resources of the node, the network transmission performance will decline due to limited forwarding resources. Therefore, it is necessary to evaluate the node resource status to prevent network congestion.

From the aspect of reliability, the above factors are combined with the status and behavior of the nodes. While ensuring that the node is not malicious, the node must complete the forwarding task quickly and efficiently. The confidentiality and integrity of data cannot guarantee the freshness of data in the network. By incorporating reliability into the trust evaluation system, the node condition can be evaluated more completely.

The node *r*_*i*_ behavior data packet *Data*_*i*_ in the SDN is represented as *Behavior Data*_*i*_, and the timestamp is appended to the end of the packet. The representation of the uploaded data packet is:

$$BehaviorData_{i}=Data_{i}\left|\left|S_{i}\right|\right|timestamp$$

$$S_{i}=SK_{i}(Data_{i})$$

Node behavior data block update algorithm process is as follows:

Algorithm 1 Node behavior data update

1. Procedure authentication (*Data*_*i*_, *PK*_*i*_)

2. *flag* = 0

3. The public key *PK*_*i*_ is an information known to all nodes, get the *PK*_*i*_ in the blockchain

4. Check the node *i* identity

5. Verify the node signature *S*_*i*_

6. If *identity*.*node* = true the node is valid.

7. Else *flag* = 1, jump to step 9

8. Forward the packet and collect the node behavior data

9. Add a new node behavior data block *BehaviorData*_*i*_ to the blockchain

10. There are some violations, the node is invalid, refuse service

11. return *flag*

12. End procedure

#### 5.1.2 Fuzzy comprehensive evaluation

In this paper, the fuzzy comprehensive evaluation method is used to evaluate the SDN nodes. The evaluation vector can not only accurately depict the object, but also further process the reference information. Because the trapezoidal and triangular membership functions are easy to calculate and consume less resource, a fuzzy subset membership function based on them with four trust levels is constructed. The result is shown in Fig 7.

**Fig 7:** Membership function.

In the third section, the entropy method is used to obtain the weight of each attribute in the node trust evaluation system. The weight of the reliability assessment attribute involves direct trust from (*w*_1_, *w*_2_, *w*_3_, *w*_4_, *w*_5_) to (*μ*_1_, *μ*_2_, *μ*_3_, *μ*_4_, *μ*_5_), and *μ*_1_ + *μ*_2_ + *μ*_3_ + *μ*_4_ + *μ*_5_ = 1. The fuzzy composition operator is used to synthesize the fuzzy weight vector and the membership matrix. The calculation process is as follows:

$$\text{B}=\text{W}\circ \text{R}=\left(\mu_{1},\mu_{2},\mu_{3},\mu_{4},\mu_{5}\right)\circ \left[\begin{array}{ccccc} r_{11} & r_{12} & r_{13} & r_{14} & r_{15}\\ r_{21} & r_{22} & r_{23} & r_{24} & r_{25}\\ r_{31} & r_{32} & r_{33} & r_{34} & r_{35}\\ r_{41} & r_{42} & r_{43} & r_{44} & r_{45}\\ r_{51} & r_{52} & r_{53} & r_{54} & r_{55} \end{array}\right]=\text{(}b_{1},b_{2},b_{3},b_{4},b_{5}),$$ (10)

In the formula 10, ∘ is a fuzzy composition operator, and *b*_*i*_ is the membership degree of fuzzy subset L in the trust evaluation of nodes. The M(·, ⊕) fuzzy composition operator not only gives consideration to the role of various factors, but also makes full use of node information. According to the definition of M(·, ⊕), the formula for *b*_*i*_ is as follow:

$$b_{i}=\text{min}(1,\sum_{i=1}^{5}\mu_{i}r_{ik}),\;k=1,2,3,4,5,$$ (11)

The weighted average principle is used to process the evaluation result vector B, and the direct trust of node *r*_*i*_ at time *t* can be expressed:

$${DTrust}_{i}(t)=\frac{\sum_{i=1}^{n}l_{i}∙a_{i}^{k}}{\sum_{i=1}^{n}a_{i}^{k}},$$ (12)

### 5.2 Indirect trust

Indirect trust is the comprehensive trust reflected by neighbor nodes. If there are malicious nodes in the SDN, they may launch selective attacks on other nodes, affecting their normal operation. The indirect trust of node *r*_*i*_ at time t can be expressed as:

$${ITurst}_{i}(t)=\frac{1}{n}\sum_{k\in C_{f}}{(DTurst}_{i,k}(t)\times {DTurst}_{k,j}(t)),$$ (13)

*C*_*f*_ represents the set of neighbor nodes after filtering, and *n* represents the number of *C*_*f*_ node sets. The SDN may contain malicious recommendation nodes. On the one hand, some nodes may give low and false recommendation value, leading to decrease the trust level of evaluated node to obtain more opportunities for data forwarding. On the other hand, some nodes may launch colluding attacks to improve their trust through high recommendation value. Therefore, the consensus mechanism of blockchain is used to filter the collected trust values.

The Proof of Work (PoW) algorithm is used to achieve consensus. By completing certain difficult computing tasks, the node which first calculates the correct answer becomes the master node, and the remaining nodes are the slave nodes. In order to reduce the time cost, when the first layer block records the node behavior, the second layer block carries out the master node election in the background. The master node generates the new block, and the slave node in turn checks whether the new block is true or not. If the master node misses signing a new block or generates a wrong block, the administrator removes its ballot and moves it out of the authorized representative list, with the remaining nodes acting as substitutes. Only when the attacker controls most nodes (51%) of the whole network, malicious nodes can implement the tampering of trust values. The specific consensus process is as follows:

1. The master node *r*_*m*_ generates a new data block and integrates its own recommended trust, attaching its digital signature and hash value of the new data block, and then broadcasts the new data block to each slave node for inspection. The new data block is expressed as:
  $${DataBlock}_{m}=(Data\_set∥Data\_hash∥{Cert}_{m}∥{Sig}_{m}∥timestamp)$$
  Data_hash=Hash(Data_set∥timestamp)
  $${Sig}_{m}={SK}_{m}(Data\_set∥Data\_hash)$$
2. After the slave node *r*_*s*_ receiving the block, it will first verify the authenticity of the block by the hash value and digital signature. If the block is illegal, the authorized representative identity of the node *r*_*m*_ will be removed and the SDN controllers will feed back to verify the node.
3. If the block is legal, the correctness of the block will be verified in the next step. Before calculating indirect trust, the value of excessive deviation will be filtered out. Set the trust value deviation *d*_*k*_. If *d*_*k*_ is large, which means the value deviates significantly from most normal values, then the recommendation trust of *r*_*s*_ is more likely to be a false value from a malicious node. After serval experiments, set deviation threshold ε = 0.1, filter out the node whose *d*_*k*_ > ε. Slave nodes will attach their digital signatures to audit results and their own recommended trust values. Then the block will broadcast to other slave nodes to realize mutual supervision and joint inspection between slave nodes.
4. After the last slave node *r*_*sn*_ receives the audit result of all other nodes, it will send a reply to the master node *r*_*m*_. The reply contains its own audit result and digital signature, all received audit results, and the conclusion. The process is expressed as:
  $${Reply}_{s}=({Data}_{s}∥{Cert}_{s}∥{Sig}_{s}∥timestamp)$$
  $${Data}_{s}=(own\_result∥receive\_result∥compare\_result)$$
  $${Sig}_{s}={SK}_{s}({Data}_{s})$$
5. The master node *r*_*m*_ summarizes the responses from all neighbor nodes. If more than 50% of the nodes agree with the legitimacy and correctness of the data block, the master node *r*_*m*_ averages all the recommended trust values received, updates the indirect trust of the node, and stores the results in the second layer of node trust data block in time sequence. The process is expressed as:
  $$DataBlock=(Data∥{Sig}_{m}∥timestamp)$$
  $$Data=(Data\_set∥Data\_hash∥{Cert}_{m}∥timestamp)$$
  $${Sig}_{m}={SK}_{m}(Data)$$
6. The master node will analyze and mark the few nodes that do not agree with the common audit results. If these nodes have malicious behaviors, the trust value of corresponding nodes will be reduced.
7. If the recommended trust value is not recognized by most of the nodes, the value is considered to be wrong and not recognized.

Node indirect trust filter algorithm process is as follows:

Algorithm 2 Node indirect trust filter

1. Procedure filter

2. *flag* = 0

3. Elect the master node *r*_*m*_ in this round

4. The master node *r*_*m*_ establishes an Indirect_trust_set

5. Sign the Indirect_trust_ set with the private key *SK*_*m*_ and broadcast it with other slave nodes (the neighbor nodes)

6.  If (authentication = = true)

7.   Proceed the Audit process

8.   *flag* = 0

9.  Else *flag* = 1

10.  The Indirect_trust_ set is valid

11.  If the indirect trust value difference between the slave node and the master node is less than 10%, attach *r*_*s*_ own indirect trust and sign it with its private key *SK*_*s*_

12.  Else the Indirect_trust_ set is invalid, mark the master node *r*_*m*_ as suspicious, alarm the SDN controller, and start the PoW algorithm to choose a new master node, jump to step 3

13.  Once all valid results from all valid nodes are gathered, the Indirect_trust_ set is confirmed as a true indirect trust value, calculate the average result

14. return *flag*

15. End procedure

### 5.3 Historical trust

In order to prevent malicious nodes from using the continuous normal behavior to quickly improve the trust value, the historical trust is introduced in the evaluation of comprehensive trust. The historical trust of node *r*_*i*_ at time *t* can be expressed:

$$HTrust_{i}(t)=\text{(}1-\lambda )HTrust_{i}(t)+\lambda HTrust_{i}\left(t-n\right),$$ (14)

*HTrust*_*i*_(t − n)is the comprehensive trust value of node *i* for the first *n* cycles. If the difference of the trust value between the before and after period is too large, the node may be considered to be untrusted. The λ is the adaptive weight of the historical trust value of the previous period, which is defined as:

$$\lambda =1-\alpha^{\frac{\Delta T}{\beta }},$$ (15)

ΔT is the difference between the trust value at the current moment and the previous period. α indicates the range of λ, β indicates the sensitivity of λ to the difference ΔT. α and β are adjustable parameters. After multiple experiments, set α = 0.95, β = 3. When the trust value of nodes increases, the growth rate of trust is slowed down to prevent malicious nodes from rapidly increasing through normal behaviors for a period of time. When the trust value of nodes decreases, the decline rate of trust will be accelerated, and the probability of untrusted nodes participating in the network will be reduced in advance.

## 6. Experimental evaluation

In order to better evaluate the effectiveness and performance of TrustBlock, Mininet and POX controller are used to conduct simulation experiments. The controller collects statistical information from the switch port, such as port number, the quantity of sent and received packets, the number of data bytes, timestamp, link status, etc., and then calculates traffic rate and link load parameters based on these information. The scene is set as follows:

Construct five management domains to simulate the network scenario of multiple SDN environments, each domain contains a controller and 40 network nodes, 1–19 malicious nodes are randomly set in each domain in the network, and selective attacks are randomly launched, which can affect the network performance. This paper does not use the standard bitcoin client, but implements a simplified version that covers the key functions of TrustBlock. The programming language used in the experiment is Python2.7.14[16] and OpenSSL 0.9.8zg [17] is used to provide the encryption library. The experimental parameters are shown in Table 1.

**Table 1:** Experiment parameters.

Parameter	Value
The total number of nodes	200
The total number of malicious nodes	1–95
Nodes transmit packet sizes	120byte
Trust renewal cycle	10min
The simulation time	2h
Initial node trust value	0.5

Considering the difference between the actual situation and the theory, the forwarding rate of the normal node cannot reach 100%. If the node is a black hole node, the forwarding rate is 0%. The initial trust value of all nodes in the SDN is 0.5. The experiment contains several iterations to simulate the continuous operation of SDN in the real scene. Two other models are compared with TrustBlock in this paper, one is a trust evaluation model based on bad behaviors (TEMBB) [18], and the other is a trust evaluation model based on bayes and risk assessment of wireless sensor networks (BRSN) [19].

### 6.1 Untrusted node identification experiment

During the simulation experiment process, the trust values of untrusted nodes and normal nodes are tested respectively under the following conditions:

1. When t = 0min to t = 30min, the node to be evaluated provides normal service, and calculating the trust value of the node.
2. When t = 30min, the untrusted node will randomly discard a part of the data packet during the forwarding process, which makes it unable to perform the following transmission, as shown in Fig 8(a).
3. When t = 30min, the untrusted node will repeat a part of the received data packets during the forwarding process, which is intended to consume network resources and reduce network lifetime, as shown in Fig 8(b).

**Fig 8:** Change trend of node trust value. **(a)** Untrust node abandons packerts randomly. **(b)** Untrust node sends packets repeatedly.

According to the experimental results, with the evaluation time gradually increases, the trust value of all nodes changes, and eventually stabilizes within a certain range. Due to different node states, the final trust value is different. As shown in Fig 8, the trust value of normal nodes increases rapidly in the first 10 cycles, and has a slower growth trend over time. The comprehensive trust of normal nodes eventually approaches 1 and stabilizes around 0.95. The trust value of untrusted nodes executing different strategies is obviously less than 1, and the final trust value is significantly lower than the initial trust value. With the increase of network running time, the decline trend tends to be flat, and finally stabilizes at about 0.3–0.4. Under the first malicious behavior strategy (Fig 8(a)), the untrusted node discards part of the data packets, so that the data cannot reach the destination host. Under the second behavior strategy (Fig 8(b)), untrusted nodes copy packets to occupy network resources, but the data can still reach the destination host. Therefore, the second behavioral strategy has a higher trust value than the first behavioral strategy, but the final trust values of both behaviors are significantly lower than the normal nodes. It can be seen from the experimental result that the TrustBlock can effectively identify the untrusted nodes in the network, and eliminate the possibility of untrusted nodes affecting the normal network communication by culling them out of the candidate forwarding nodes.

### 6.2 Trust value impact factor assessment

In order to prove that the method proposed in this paper based on three-dimensional factors (i.e. direct trust, indirect trust and historical trust) is superior to the direct trust evaluation method, the two methods are compared. The simulation results are shown in Fig 9.

**Fig 9:** Trust values of nodes in different evaluation methods. **(a)** Normal node evaluation factor impact. **(b)** Untrust node evaluation factor impact.

By analyzing the experimental results, it can be seen from Fig 9(a) that, when evaluating the trust of normal nodes, the trust calculation method based on three-dimensional factors is approximate to the final value obtained by using the direct trust calculation method. However, TrustBlock can slow down the rising rate of trust by combining historical trust and effectively prevent untrusted nodes from rapidly improving their trust value through normal behaviors over a period of time. It can be seen from Fig 9(b) that, compared with the direct trust value assessment only, the three-dimensional factors method makes the trust value decline faster, and the trust value of the untrusted node is lower in the final state. TrustBlock gives more comprehensive consideration to the trust state of nodes, and can distinguish normal nodes from untrusted nodes more quickly and effectively.

### 6.3 Anti-periodic attack experiment

In the real life, untrusted nodes may improve their trust value by periodic normal behaviors. Assume that the untrusted node appears as a normal node in the first 6 cycles, becomes a malicious node in 7–12 cycles, and randomly discards data packets or forwards duplicate data at a forwarding rate of 0.3 to 0.6. The attack was stopped at 13 cycles, which makes it performance as a normal node, and then appeared as a malicious node at 18 cycles. The change trend of the trust value is shown in Fig 10.

**Fig 10:** Change trend of node trust value during periodic attacks.

It can be seen from Fig 10 that the TrustBlock can effectively resist the periodic attack. By comparing the difference between current trust and historical trust, TrustBlock effectively slows down the rise of node trust and speeds up the decline of node trust. When a node launches an attack, it needs to ensure a high-quality data forwarding service for a long period of time to maintain its trust level within the normal node. When the node behavior begins to be untrustworthy, the node trust value drops rapidly. TrustBlock implements the forwarding task by using a highly trusted node, so that the SDN controller can exclude the untrusted node from the candidate forwarding set as soon as possible, which can effectively improve the forwarding efficiency of the SDN.[20]

### 6.4 Anti-collusion attack experiment

By providing false recommendation trust values, malicious nodes defame other nodes and reduce the average trust level of normal nodes. Or malicious nodes can directly improve their trust level through collusion attack. This paper realizes the filtering of false recommendation values through the blockchain consensus mechanism, reduces the impact of dishonest recommended trust values, and further monitors the nodes through the blockchain. Conduct anti-collusive attack experiment, neighbor nodes only provide false recommendation trust value, and do not conduct other attacks. Set the malicious recommendation rate of 0.1–0.3, perform iterative experiments, and observe the influence of collusive attacks on indirect trust and the defense capability of TrustBlock.

As shown in Fig 11, in the colluding attack experiment, untrusted nodes randomly provide false recommendation values. With the increase of the proportion of malicious nodes, the gap between the value obtained by TrustBlock and the actual value gradually increases, but it still remains within a certain range with a small precision loss. But the TEMBB and BRSN algorithms are greatly affected by the untrusted node, which may lead to deviations in the final evaluation result. TrustBlock can effectively implement the filtering of recommended values through the consensus mechanism. At the same time, with PoW algorithm, false recommendation will be recognized only if more than 1/2 nodes are controlled. Once the false recommendation behavior is found, SDN controller can use the traceability of blockchain to focus on the nodes and reduce the trust value of them.

**Fig 11:** Malicious recommendation value filtering. **(a)** Normal node indirect trust value filtering. **(b)** Untrust node indirect trust value filtering.

### 6.5 TrustBlock detection accuracy analysis

This paper uses four basic metrics True Positive (TP), True Negative (TN), False Positive (FP), and False Negative (FN) to construct four metrics: Detection Rate (*DR*), True Positive Rate (*TPR*), False Positive Rate (*FPR*), and Accurate Rate (*AR*) to evaluate the scheme in this paper, and the results are evaluated from the following aspects:

$$DR=\frac{TP}{TP+FP},$$ (16)

$$TPR=\frac{TP}{TP+FN},$$ (17)

$$FPR=\frac{FP}{TN+FP},$$ (18)

$$AR=\frac{TP+TN}{TP+FP+TN+FN},$$ (19)

The indicators are DR(the model predicts the correct proportion of all results), TPR (the ratio of correctly true samples in all samples which were actually true), FPR(the ratio that was falsely judged to be true in all samples which were actually false) and AR(the proportion of correct predictions). Where TP represents the number of untrusted nodes marked correctly, FP represents the number of untrusted nodes marked incorrectly, TN represents the number of trusted nodes marked correctly, and FN represents the number of trusted nodes marked incorrectly. When the DR, TPR, AR metrics are high, and the FPR is low, it can reflect that the model has better performance. The results are shown in Fig 12.

**Fig 12:** TrustBlock detection rate analysis.

Comparing the analysis results with the TEMBB and BRSN evaluation model, it can be seen that the detection rate and accuracy of the TrustBlock are the highest, and the false positive rate is the lowest. And TrustBlock filters the malicious recommendation trust value, which can resist the collusion attack more intelligently. The positive sample recall rate is the highest and the negative sample judgment error rate is much lower than other models. It proves that the TrustBlock method is effective and can detect the trust state of nodes in the network more accurately.

On this basis, the variation of detection accuracy with the number of untrusted nodes is considered respectively:

1. When the total number of nodes is fixed (200) and the number of untrusted nodes gradually increases (no more than 25%), the detection rate changes with the number of untrusted nodes.
2. When the ratio of the untrusted nodes to the total number of network nodes is fixed (20%), the detection rate changes as the total number of nodes increases.

As shown in Fig 13, TrustBlock detection accuracy is about 97.8% under normal circumstances. When the total number of untrusted nodes in SDN is fixed and the number of untrusted nodes increases, the detection accuracy of nodes has a downward trend, but remains at 93%, which can still accurately detect untrusted nodes in the network. When the density of untrusted nodes is fixed and the total number of nodes keeps increasing, the detection accuracy of nodes decreases more gently than before, remaining at about 95%. TrustBlock can more conveniently screen untrusted nodes through blockchain, and guarantee the traceability and authenticity of node behaviors through behavioral data blocks. Nodes cannot deny the behaviors that have occurred, which can reduce the detection error rate. It can be seen from the above analysis that TrustBlock is less affected by untrusted nodes and more stable.

**Fig 13:** Detection accuracy rate changes with untrusted nodes.

### 6.6 Network performance change experiment

The purpose of TrustBlock is to select more secure and reliable nodes for data transmission. Based on this, the performance change of SDN is analyzed, including the change of network throughput (Fig 14) with the increase of untrusted nodes.

**Fig 14:** Trends in network throughput of untrusted nodes increasing.

Due to the selective attack of malicious nodes, the data transmission failure will lead to the decline of SDN throughput, and the data repeated transmission caused by packet loss will lead to the increase of the end-to-end delay of SDN. With the increase of untrusted nodes in the network, the throughput of existing routing algorithms will decline rapidly due to the lack of node trust evaluation mechanism. In this paper, trust is taken as the security attribute of routing partition, which can effectively detect untrusted nodes and filter the nodes in the candidate forwarding set, select more secure and reliable nodes for data transmission, and maintain the stability of the SDN. TrustBlock reduces the network node packet loss rate caused by untrusted nodes, which increases the throughput of the entire network, and end-to-end delay is also more stable.

## 7. Conclusions

A TrustBlock method is purposed in this paper, which calculates the trust value of SDN node based on blockchain. First, the weights of each evaluation attribute are determined by the entropy method. Then, from the perspective of direct trust, indirect trust and historical trust, the comprehensive trust value of the node is calculated. In the process of calculation, the forwarding state is used to evaluate the node reliability, and the blockchain is used to realize the identity authentication. The fuzzy comprehensive evaluation model is used to calculate the trust value. In the process of indirect trust calculation, the consensus mechanism of blockchain is used to achieve the filtering of malicious recommendation nodes. In the process of historical trust calculation, the adaptive history trust weight is used to prevent the trust value from rising too fast. The blockchain is used to store trust values, which guarantees the data authenticity, irreparability and openness. The simulation results show that compared with other models, the detection rate reaches 98.8%, and the accuracy rate reaches 98%. Therefore, the trust evaluation method called TrustBlock proposed in this paper can detect node trust status in the network more accurately. To evaluate the node status, the interaction risk between nodes can be reduced, and the robustness of the SDN system can enhance.

Although a SDN node trust evaluation model is established in this paper, there are still some shortcomings about it. This paper establishes a node trust evaluation system based on node behavior and node status from two aspects of security and reliability. But, the premise of the system is that there are a lot of interactions in the SDN and the nodes can learn from each other. However, in cases where there is less network activity during the application, a mechanism is needed to proactively establish trust between nodes. For example, a guiding mechanism that uses trusted nodes as a trust base can be established, and the trusted node actively generates some events in the network to provide nodes with opportunities to supervise and learn from each other. In general, the trust problem of SDN nodes is a complex research problem, which needs to be studied from many aspects. This article only provides a way of thinking and a theory to solve the trust problem of SDN. In future work, more in-depth research is needed.

## Supporting information

S1 Data (CSV)
